The article "Ethanol Extract of Sargassum siliquastrum Inhibits Lipopolysaccharide-Induced Nitric Oxide Generation by Downregulating the Nuclear Factor-Kappa B Signaling Pathway" was published in 2022. Journal: Evid Based Complement Alternat Med.

# Ethanol Extract of *Sargassum siliquastrum* Inhibits Lipopolysaccharide-Induced Nitric Oxide Generation by Downregulating the Nuclear Factor-Kappa B Signaling Pathway

**DOI:** 10.1155/2022/6160010

**Published:** 2022-06-10

**Authors:** Hye-Young Min, Hyewon Kim, Ho Jin Lee, Na-Young Yoon, Yeon-Kye Kim, Ho-Young Lee

**Affiliations:** ^1^College of Pharmacy and Research Institute of Pharmaceutical Sciences, Seoul National University, Seoul 08826, Republic of Korea; ^2^Division of Food Safety and Processing Research, National Institute of Fisheries Science, Busan 46083, Republic of Korea

## Abstract

*Sargassum siliquastrum* (SS) is an edible brown seaweed widely consumed in Korea and considered a functional food source. Previous studies have reported various biological activities of SS extracts, including antioxidant and hepatoprotective properties. In the present study, we examined the anti-inflammatory effects of the SS extract and assessed the underlying mechanism of action. The SS extract significantly inhibited lipopolysaccharide (LPS)-induced nitric oxide (NO) production in a dose-dependent manner (% of NO production at 500 *μ*g/mL: 60.1 ± 0.9%), with no obvious toxicity. Furthermore, the SS extract inhibited mRNA and protein expression levels of inducible NO synthase, as well as LPS-induced expression and production of proinflammatory cytokines such as IL-1*β*, IL-6, or TNF-*α* (IL-6 production (ng/mL) : LPS−: 0.7 ± 0.3; LPS+: 68.1 ± 2.8; LPS + SS extract: 51.9 ± 1.2; TNF-*α* production (ng/mL) : LPS−: 0.3 ± 0.1; LPS+: 23.0 ± 0.1; LPS + SS extract: 18.2 ± 10.8). Mechanistically, the SS extract attenuated LPS-induced activation of the nuclear factor kappa-light-chain-enhancer of activated B cells (nuclear factor-kappa B, NF-*κ*B) signaling pathway such as phosphorylation of NF-*κ*B p65 and degradation of I*κ*B-*α*, thereby blocking LPS-induced activation of NF-*κ*B transcriptional activity. The SS extract also enhanced LPS-induced heme oxygenase-1 expression and attenuated LPS-induced cellular reactive oxygen species production (% of ROS production at 500 *μ*g/mL: 52.2 ± 1.3%). Collectively, these findings suggest that the SS extract elicits anti-inflammatory effects in mouse macrophage cells.

## 1. Introduction

Despite the crucial role of inflammation in host defense against various insults, deregulation of inflammatory processes can seriously impact the resolution of inflammation and promote chronic inflammation [1, 2]. Given the involvement of chronic inflammation in several pathological conditions, including metabolic syndromes, cardiovascular diseases, autoimmune diseases, and cancer [1], suppression of excessive inflammatory responses is required to maintain homeostasis and treat inflammatory diseases.

The article "Ethanol Extract of Sargassum siliquastrum Inhibits Lipopolysaccharide-Induced Nitric Oxide Generation by Downregulating the Nuclear Factor-Kappa B Signaling Pathway" was published in 2022. Journal: Evid Based Complement Alternat Med.

Nitric oxide (NO) is closely associated with various pathophysiological conditions, including inflammation, immunity, and cancer [3, 4]. NO is a byproduct produced by the conversion of L-arginine to citrulline by three isoforms of NO synthase (NOS), either constitutive (neuronal NOS (nNOS) and endothelial NOS (eNOS)) or inducible (iNOS) forms [3]. eNOS and nNOS regulate tissue homeostasis such as vasodilation [3, 5], whereas iNOS plays an important role in various inflammatory responses [3]. iNOS expression is transcriptionally regulated in response to various proinflammatory inducers [3, 6]. For example, bacterial glycolipid lipopolysaccharide (LPS) binds to toll-like receptor 4 (TLR4) and activates downstream signaling cascades, such as the MyD88-dependent TIRAP/TRAF6/TAK1 and the MyD88-independent TRAM/TRIF/TBK1/IRF3 pathway [7, 8]. TAK1 further phosphorylates either the I*κ*B kinase complex (IKK*α*/*β*) or mitogen-activated protein kinases (MAPKs; JNK, ERK, and p38 MAPK), eventually activating nuclear factor kappa-light-chain-enhancer of activated B cells (nuclear factor-kappa B, NF-*κ*B) and activator protein-1 (AP-1) and inducing various inflammation-associated target genes, including iNOS [8, 9]. iNOS has been implicated in infectious and inflammatory diseases, neurodegenerative disorders, cancer, and pulmonary emphysema [10–12], and pharmacological blockade of iNOS has been shown to inhibit tumor growth [13], enhance the efficacy of antitumor immunotherapies [14], and ameliorate elastase-induced pulmonary emphysema and pulmonary hypertension [15]. These findings indicate that iNOS may be a potential target for treating various inflammation-associated disorders.

The heme oxygenase pathway plays an important role in maintaining homeostasis by acting as a sensor of cellular oxidative stress [16]. Heme oxygenases catalyze heme degradation into carbon monoxide, ferrous iron, and bilirubin [16]. Two isoforms of heme oxygenases, i.e., the inducible (HO-1) and constitutively expressed (HO-2) forms, have been identified [16]. HO-1 is induced by various transcription factors, including nuclear factor-erythroid factor 2-related factor 2 (Nrf2), which exerts antioxidant, anti-inflammatory, and antiapoptotic activities [16, 17]. Induction of heme oxygenase-1 (HO-1) reduces LPS-induced NO production and iNOS expression by downregulating iNOS activity as well as NF-*κ*B pathway activation [18]. Therefore, agents that are able to modulate the Nrf2/HO-1 pathway exert anti-inflammatory action through disrupting the NF-*κ*B/iNOS pathway.

Edible seaweeds contain various nutrients and have been utilized as functional foods and complementary therapies [19, 20]. The brown seaweed *Sargassum* species has been utilized in traditional medicine and reportedly exerts antioxidant, anti-inflammatory, antiviral, and anticancer activities [21, 22]. *Sargassum siliquastrum* (SS) is a Korean indigenous brown alga belonging to the Sargassaceae family [23, 24]. SS extracts are known to exert several biological activities, including antioxidant effects and protection against carbon tetrachloride-induced hepatic injury [23, 24]. In the present study, we examined the anti-inflammatory effect of the methanol extract of SS and investigated its underlying mechanism of action.

The article "Ethanol Extract of Sargassum siliquastrum Inhibits Lipopolysaccharide-Induced Nitric Oxide Generation by Downregulating the Nuclear Factor-Kappa B Signaling Pathway" was published in 2022. Journal: Evid Based Complement Alternat Med.

## 2. Materials and Methods

### 2.1. Reagents

Dulbecco's modified Eagle medium (DMEM), fetal bovine serum (FBS), phosphate-buffered saline, and antibiotic-antimycotic solution were purchased from Welgene Inc. (Gyeongsan-si, Gyeongsangbuk-do, Republic of Korea). Antibodies against phosphorylated p42/p44 MAPK (pERK1/2, T202/Y204), phosphorylated Akt (pAkt, S473), Akt, and phosphorylated c-Jun (p-c-Jun, S63) were purchased from Cell Signaling Technology (Danvers, MA, USA). Antibodies against phosphorylated NF-*κ*B p65 (pp65, S536), NF-*κ*B p65, I*κ*B-*α*, ERK1, c-Jun, phosphorylated p38 (pp38, Y182), p38, JNK1, c-Jun, and *β*-actin were purchased from Santa Cruz Biotechnology (Dallas, TX, USA). A primary antibody against iNOS was purchased from Abcam (Cambridge, UK). A primary antibody against HO-1 was purchased from Enzo Life Sciences (Farmingdale, NY, USA). LPS, crystal violet, and other chemicals were purchased from Sigma-Aldrich (St. Louis, MO, USA) unless otherwise specified.

### 2.2. Preparation of SS Extract

SS was collected from the coast of Tongyeong si (Gyeongsangnam-do, Republic of Korea) in 2020 and stored in a freezer at –20°C until use. A voucher specimen (no. KGTS-29) was deposited at the National Institute of Fisheries Science Laboratory. Frozen SS (10 g) was extracted with 75% ethanol three times at room temperature for 3 h. The yield of the extract was 5.94%. The crude extract was dissolved in sterile deionized water and used for in vitro experiments.

### 2.3. Cell Culture

Mouse macrophage RAW 264.7 cells were kindly provided by Dr. Sang Kook Lee (Seoul National University, Seoul, Republic of Korea). RAW 264.7 cells were maintained in DMEM supplemented with 10% FBS and antibiotics (100 units/mL penicillin, 100 *μ*g/mL streptomycin sulfate, and 250 ng/mL amphotericin B in 0.85% NaCl solution). The cells were incubated at 37°C with 5% CO_2_ in a humidified atmosphere.

### 2.4. Nitrite Assay

The nitrite assay was performed as described previously [25]. In brief, RAW 264.7 cells were plated in 24-well plates (2.5 × 10^5^ cells/well) and incubated for 24 h. Then, the culture media was replaced with fresh media, and cells were stimulated with 1 *μ*g/mL LPS in the presence or absence of the SS extract. After an additional 20 h, the media was collected, and 50 μL of the media was incubated with 50 *μ*L of 1% sulfanilamide solution (dissolved in 5% H_3_PO_4_) in 96-well plates. After incubation for 10 min at room temperature, 50 *μ*L of 0.1% N-1-naphthylethylenediamine dihydrochloride solution was added, and the absorbance was measured at 540 nm. The nitrite concentration was determined by comparing a standard sodium nitrite curve.

The article "Ethanol Extract of Sargassum siliquastrum Inhibits Lipopolysaccharide-Induced Nitric Oxide Generation by Downregulating the Nuclear Factor-Kappa B Signaling Pathway" was published in 2022. Journal: Evid Based Complement Alternat Med.

### 2.5. Cell Viability Assay

The cytotoxicity of the SS extract was determined under the same experimental conditions as the nitrite assay (treatment with the SS extract for 20 h). In order to perform a crystal violet assay [26], the remaining cells after media collection were fixed with 100% methanol for 30 min at room temperature and air-dried. Fixed cells were stained with 0.025% crystal violet solution for 30 min at room temperature and then washed multiple times with tap water. Stained cells were dissolved in 1% sodium dodecyl sulfate (SDS) solution, and the absorbance was measured at 570 nm. Cell viability was determined by comparing with LPS-stimulated control cells. A CCK-8 assay [27] was performed according to the manufacturer's provided protocol. In brief, cells were seeded into 96-well plates (5 × 10^4^ cells/well) and incubated for 24 h. Cells were treated with the SS extract for 20 h. After the drug treatment, the cells were treated with the CCK-8 solution (10 *μ*L per well) and then incubated for 2 h in the CO_2_ incubator. The absorbance was measured at 450 nm. Cell viability was determined by comparison with the vehicle (water) treated control cells.

### 2.6. Western Blot Analysis

Western blot analysis was performed as described previously [28]. In brief, RAW 264.7 cells were stimulated with LPS (1 *μ*g/mL) in the absence or presence of the SS extract for 20 h. To determine the effect of the SS extract on LPS-induced activation of the TLR4 pathway, cells were pretreated with the SS extract for 24 h and then stimulated with LPS (1 *μ*g/mL) for 30 min. Total cell lysates were prepared with RIPA buffer (50 mM tris-HCl (pH 7.4), 150 mM NaCl, 1% Triton X-100, 0.25% sodium deoxycholate, 1 mM EDTA) containing protease and phosphatase inhibitors. The protein concentration was determined using a BCA assay kit (Thermo Fisher Scientific, Waltham, MA, USA). Equal amounts of protein (20–25 *μ*g) were subjected to 9% sodium dodecyl sulfate-polyacrylamide gel electrophoresis (SDS-PAGE) and transferred onto polyvinylidene difluoride (PVDF) membranes (ATTO Corp., Tokyo, Japan). Membranes were incubated with blocking buffer (5% nonfat dry milk in tris-buffered saline (TBS) containing 0.01% Tween-20 (TBST)) for 1 h at room temperature and then incubated with primary antibodies diluted in 3% bovine serum albumin in TBST (1 : 1,000) overnight at 4°C. Membranes were washed three times with TBST and incubated with secondary antibodies diluted in 3% nonfat dry milk in TBST (1 : 5,000) for 1 h at room temperature. The membranes were washed multiple times with TBST, and protein bands were visualized using an enhanced chemiluminescence (ECL) detection kit (Thermo Fisher Scientific). Densitometric analysis was performed using ImageJ software (version 1.51j8, National Institutes of Health, Bethesda, MA, USA). The band intensity of each marker was expressed as relative protein expression (densitometry of each marker normalized to loading control protein (*β*-actin)).

The article "Ethanol Extract of Sargassum siliquastrum Inhibits Lipopolysaccharide-Induced Nitric Oxide Generation by Downregulating the Nuclear Factor-Kappa B Signaling Pathway" was published in 2022. Journal: Evid Based Complement Alternat Med.

### 2.7. Real-Time PCR

Real-time PCR was performed as described previously [29]. In brief, RAW 264.7 cells were stimulated with 1 *μ*g/mL LPS with or without the SS extract for 20 h. Total cellular RNA was isolated using a phenol-chloroform extraction method, reverse transcribed using a first-strand cDNA synthesis kit (TransGen, Beijing, China) and analyzed by real-time PCR with SYBR green-based qPCR master mix solution (Enzynomics, Daejeon, Korea) and gene-specific primers (COSMO Genetech, Inc., Seoul, Republic of Korea; listed in Table 1). The thermocycler conditions were as follows: preincubation at 95°C for 10 min; 50 cycles of 95°C for 10 s, 60°C for 26 s; melting curve analysis was performed to determine reaction specificity. Gene expression was determined using the 2^−ΔΔCt^ method as described previously [30]. 18S rRNA was used as a reference gene.

### 2.8. Measurement of Interleukin-6 (IL-6) and Tumor Necrosis Factor-Alpha (TNF-*α*) Production

The effects of the SS extract on LPS-induced IL-6 and TNF-*α* production were determined using commercially available ELISA kits (R&D systems, Minneapolis, MN) according to the protocol provided by the manufacturer. The culture media, obtained from the same experimental conditions as the nitrite assay, were used for ELISA.

### 2.9. Reporter Gene Assay

In brief, RAW 264.7 cells were seeded in a 24-well plate and transiently transfected with 3 × *κ*B-Luc vector (a gift from Dr. Denis C. Guttridge, Medical University of South Carolina, SC, USA) [31]], the Col-Z-Luc vector [32], or the Nrf2-Luc vector (a gift from Dr. Mi-Kyoung Kwak, College of Pharmacy, Catholic University, Bucheon-si, Gyeonggi-do, Republic of Korea) [33] in the presence of pCMV-*β*-gal using Lipofectamine^™^ Reagent with PLUS^™^ Reagent (Thermo Fisher Scientific) according to the manufacturer's instructions. Cells were stimulated with LPS (1 *μ*g/mL) in the absence or presence of the SS extract for 6 h. Then, cells were lysed with 1× lysis juice (PJK GmbH, Kleinblittersdorf, Germany). Luciferase reporter activity was determined using the beetle-juice luciferase assay kit (PJK GmbH) and normalized to *β*-galactosidase activity determined using *β*-gal juice (PJK GmbH).

The article "Ethanol Extract of Sargassum siliquastrum Inhibits Lipopolysaccharide-Induced Nitric Oxide Generation by Downregulating the Nuclear Factor-Kappa B Signaling Pathway" was published in 2022. Journal: Evid Based Complement Alternat Med.

### 2.10. Measurement of the Cellular Reactive Oxygen Species (ROS) Production

Cellular ROS levels were determined using a 2',7'-dichlorodihydrofluorescein diacetate (H_2_DCFDA) probe as described previously [28]. Cells were seeded into 96-well plates in black with a clear bottom (5 × 10^4^ cells/well) and incubated for 24 h. Cells were stimulated with LPS (1 *μ*g/mL) in the absence or presence of the SS extract for 20 h. After the drug treatment, the cells were treated with the H_2_DCFDA solution (final 20 *μ*M) and then incubated for 1 h in the CO_2_ incubator. Fluorescence was measured using a SpectraMax M5 multimode microplate reader (Molecular Devices, San Jose, CA, USA) at an excitation wavelength of 485 nm and an emission wavelength of 535 nm.

### 2.11. Statistical Analysis

Data were analyzed using GraphPad Prism 9 (GraphPad Software, Inc., La Jolla, CA, USA). Data values are presented as the mean ± standard deviation (SD), and statistical significance of differences was determined using one-way analysis of variance (ANOVA), followed by Dunnett's multiple comparison test for comparison with the indicated group. Statistical significance was set at *p* < 0.05.

## 3. Results

### 3.1. SS Extract Efficiently Inhibits LPS-Induced NO Production without Toxicity

We evaluated the effect of the SS extract on LPS-induced NO production in mouse macrophage RAW 264.7 cells, stimulating cells with LPS in the absence or presence of the SS extract. The SS extract inhibited LPS-induced NO production in a dose-dependent manner (Figure 1(a)). In addition, no morphological changes related to cell death, such as increases in cell debris and floating cells, were observed in cells treated with the SS extract. Therefore, to precisely determine whether these effects were due to cytotoxicity of the SS extract, we performed cell viability assays (a crystal violet assay and a CCK-8 assay) under the same experimental conditions as the nitrite assay. Under experimental conditions, the SS extract demonstrated no cytotoxicity toward macrophages (Figure 1(b)), suggesting that the inhibitory effect of the SS extract on LPS-induced NO production could not be attributed to cytotoxicity. These results suggest the suppressive effect of the SS extract on LPS-induced NO production with no overt toxicity.

The article "Ethanol Extract of Sargassum siliquastrum Inhibits Lipopolysaccharide-Induced Nitric Oxide Generation by Downregulating the Nuclear Factor-Kappa B Signaling Pathway" was published in 2022. Journal: Evid Based Complement Alternat Med.

### 3.2. SS Extract Downregulates LPS-Induced iNOS Expression

Given the efficient inhibitory effects of the SS extract on LPS-induced NO production, we next examined the effects of this extract on LPS-induced iNOS mRNA and protein expression. The SS extract significantly ameliorated the LPS-induced increase in *Nos2* expression in mouse macrophage cells (Figure 2(a)). Consistently, the SS extract markedly attenuated the LPS-induced increase in iNOS protein expression (Figure 2(b)). These results indicate that the SS extract inhibits LPS-induced NO production by downregulating iNOS protein and mRNA expression in mouse macrophage cells.

### 3.3. SS Extract Inhibits LPS-Induced Proinflammatory Cytokine Expression and Production

As the SS extract markedly suppressed LPS-induced iNOS expression, we examined the inhibitory effects of this extract on LPS-induced proinflammatory cytokine expression in mouse macrophage cells. We observed that the SS extract efficiently inhibited the LPS-induced increase in *Il1b* (encoding IL-1*β*), *Il6* (encoding IL-6), and *Tnf* (encoding TNF-*α*) expression in mouse macrophage cells (Figure 3(a)). The SS extract also inhibited LPS-induced IL-6 and TNF-*α* production in mouse macrophage cells (Figure 3(b)). These results indicate the anti-inflammatory effect of the SS extract in mouse macrophage cells.

### 3.4. SS Extract Decreases LPS-Mediated Activation of NF-*κ*B but Not AP-1

We further examined the effects of the SS extract on LPS-mediated activation of the TLR4 signaling pathway. We first validated LPS-induced NF-*κ*B or MAPK pathway activation using known inhibitors, such as BAY 11–7082 (BAY, an IKK/NF-*κ*B inhibitor [34]), U0126 (U, a MEK/ERK inhibitor [35]), SP600125 (SP, a JNK inhibitor [36]), and SB203580 (SB, a p38 MAPK inhibitor [37]) using respective markers (phosphorylated NF-*κ*B p65 (S536), a target protein for IKK [38], for BAY 11–7082; phosphorylated ERK1/2 for U0126; phosphorylated JNK1/2 for SP600125; and phosphorylated CREB, a target protein for p38 MAPK [39], for SB203580). Stimulation of RAW 264.7 cells with LPS for 30 min upregulated the phosphorylation of a downstream target of IKK*α*/*β*, such as NF-*κ*B p65 (Figure 4(a)). In addition, LPS stimulation increased the phosphorylation of ERK, JNK, and CREB, a downstream target of p38 MAPK (Figure 4(a)). These events were markedly suppressed by treatment with the specific inhibitors (Figure 4(a)). We then examined the effect of the SS extract on LPS-induced activation of NF-*κ*B and MAPK pathways. Treatment with the SS extract attenuated LPS-induced phosphorylation of NF-*κ*B p65 and degradation of I*κ*B-*α* (Figure 4(b)). However, the SS extract minimally affected the LPS-mediated increased phosphorylation of ERK, p38 MAPK, JNK, and the downstream c-Jun (Figure 4(c)). Consistent with the decreased p65 phosphorylation following treatment, the SS extract suppressed LPS-induced NF-*κ*B transcriptional activity in RAW 264.7 cells (Figure 4(d)). These results suggest that the SS extract suppresses LPS-induced iNOS expression by downregulating NF-*κ*B activation in RAW 264.7 cells.

The article "Ethanol Extract of Sargassum siliquastrum Inhibits Lipopolysaccharide-Induced Nitric Oxide Generation by Downregulating the Nuclear Factor-Kappa B Signaling Pathway" was published in 2022. Journal: Evid Based Complement Alternat Med.

### 3.5. SS Extract Enhances LPS-Induced HO-1 Expression

Based on the role of the Nrf2/HO-1 pathway in the negative regulation of LPS-mediated NF-*κ*B/iNOS pathway activation [18], we further examined the effect of the SS extract on the activation of the Nrf2/HO-1 pathway. Because Nrf2 is known to be activated by the PI3K/Akt pathway [40] and LPS activates the PI3K/Akt pathway [41], we investigated the effect of the SS extract on the activation of the PI3K/Akt/Nrf2 pathway by determining the level of phosphorylated Akt and HO-1 expression as indicators of the pathway activation. We observed that treatment with the SS extract alone minimally affected Akt phosphorylation and HO-1 expression in macrophage cells (Figure 5(a)). However, despite having a minimal effect on LPS-induced Akt activation, the SS extract increased the LPS-induced HO-1 expression in macrophage cells (Figure 5(a)). In addition, the SS extract also enhanced LPS-induced increases in *Hmox1* (encoding HO-1) mRNA expression (Figure 5(b)) and the Nrf2 reporter activity (Figure 5(c)) in macrophage cells. These results indicate that the SS extract enhances LPS-induced activation of the Nrf2/HO-1 pathway. Based on the activation of Nrf2 by oxidative stress [18, 42] and LPS as a ROS inducer in macrophages [43], we further determined whether the SS extract could modulate LPS-induced oxidative stress in macrophages. We observed that stimulation with LPS markedly elevated cellular ROS levels, which was significantly attenuated by treatment with the SS extract in macrophage cells (Figure 5(d)). These results suggest that modulation of the ROS/Nrf2 pathway might be involved in the anti-inflammatory effect of the SS extract in macrophage cells.

### 3.6. Fatty Acid Contents of the SS Extract

Based on the health benefits of bioactive fatty acids through modulation of immune function and alleviation of inflammation [44], we additionally determined the level of various fatty acids in the SS extract. We found that, in addition to saturated fatty acids, the SS extract contains various mono- or polyunsaturated fatty acids (PUFAs), such as cis-4, 7, 10, 13, 16, 19-docosahexaenoic acid (DHA) and cis-5, 8, 11, 14, 17-eicosapentaenoic acid (EPA) (Table 2).

The article "Ethanol Extract of Sargassum siliquastrum Inhibits Lipopolysaccharide-Induced Nitric Oxide Generation by Downregulating the Nuclear Factor-Kappa B Signaling Pathway" was published in 2022. Journal: Evid Based Complement Alternat Med.

## 4. Discussion

In the present study, we demonstrated the inhibitory effect of the SS extract on LPS-induced iNOS expression. Based on our findings, the SS extract induced NO production by downregulating iNOS mRNA and protein expression with no significant toxicity under the experimental conditions. Furthermore, the SS extract inhibited the LPS-induced increase in proinflammatory cytokine expression. Mechanistically, the SS extract inhibited LPS-induced activation of the NF-*κ*B signaling pathway such as phosphorylation of NF-*κ*B p65 and degradation of I*κ*B-*α*, thereby disrupting the LPS-induced activation of NF-*κ*B transcriptional activity (Figure 5(e)). The SS extract also enhanced LPS-induced HO-1 expression and attenuated LPS-induced cellular reactive oxygen species production (Figure 5(e)). These findings suggest that SS extract has anti-inflammatory effects in mouse macrophage cells.

Edible marine products with biological functions have been utilized as functional foods and complementary and alternative medicines. In addition, similar to the successful development of therapeutic agents from plant-derived natural products [45], marine natural products are considered important sources for drug development [46]. Therefore, identifying the biological effects of marine natural products is pivotal for developing novel therapeutic and preventive regimens. In the present study, we demonstrated the anti-inflammatory effects of the SS methanol extract on murine macrophage cells, mediated by downregulating iNOS expression by suppressing NF-*κ*B and enhancing LPS-mediated HO-1 induction. Inflammation, particularly low levels of chronic inflammation, is closely involved in various pathological disorders [1]. Among several inflammation-associated enzymes, iNOS has been implicated in various chronic progressive diseases, including autoimmune diseases, cancer, and pulmonary emphysema [10,11]. In addition, NF-*κ*B is a key transcription factor involved in the transcription of various proinflammatory cytokines, chemokines, and other inflammation-associated factors [47]. The Nrf2/HO-1 pathway inhibits inflammation by interfering with the NF-*κ*B pathway and its downstream target proteins in a functional or transcriptional manner [18]. Hence, agents that can inhibit iNOS expression or modulate the Nrf2/HO-1 pathway could be potential candidates for developing efficacious therapeutic agents against inflammation-associated chronic diseases. Collectively, the present results suggest the potential utility of the SS extract as complementary medicine, functional food, or adjuvant therapy for the treatment of chronic inflammatory disorders, including pulmonary emphysema.

The article "Ethanol Extract of Sargassum siliquastrum Inhibits Lipopolysaccharide-Induced Nitric Oxide Generation by Downregulating the Nuclear Factor-Kappa B Signaling Pathway" was published in 2022. Journal: Evid Based Complement Alternat Med.

Although this study demonstrated the anti-inflammatory effect of the SS extract, previous studies have demonstrated the biological effects of several constituents of SS. For instance, SS-derived fucoxanthin exerted cytoprotective effects against hydrogen peroxide or UV-induced cell damage [48, 49] and matrix metalloproteinase expression in fibrosarcoma cells [50]. In addition, SS-derived farnesylacetones exhibit a vasodilatory effect [51]. Moreover, meroterpenoids displayed antioxidant effects [52] cytotoxicity in human cancer cells [53], and the meroterpenoid, sargachromanol G, exhibited anti-inflammatory effects in mouse macrophage cells [54]. Therefore, the anti-inflammatory effect of the SS extract might be due to the anti-inflammatory effect mediated by sargachromanol G. In addition, we found that the SS extract contains various PUFAs. These PUFAs have been known to possess strong anti-inflammatory effects and have been widely utilized as nutraceuticals [55]. Thus, although additional investigation should be required, these PUFAs might play a role in the anti-inflammatory activity of the SS extract in macrophage cells. Further studies are required to identify additional active compounds exerting the anti-inflammatory effects of SS. In addition, the inhibitory effect of previously identified SS-derived compounds on LPS-mediated inflammatory processes needs to be examined in future studies.

## 5. Conclusions

The present study demonstrates the anti-inflammatory effect of the SS extract, mediated by downregulating the NF-*κ*B-mediated expression of proinflammatory mediators. Further studies are warranted to investigate additional biological activities of the SS extract and the underlying mechanism of action and to identify active principal compounds using additional and advanced preclinical settings.

## Figures and Tables

**Figure 1:** SS extract suppresses LPS-induced NO production without toxicity. (a) Effects of the SS extract (SS) on LPS-induced NO production, determined by the nitrite assay. (b) Cytotoxicity of the SS extract (SS) in RAW 264.7 cells under experimental conditions identical to the nitrite assay. Cytotoxicity was determined by the crystal violet (left) and the CCK-8 (right) assays. The bars represent the mean ± standard deviation (SD). ^∗^: *P* < 0.05, ^∗∗^: *P* < 0.01, and ^∗∗∗^: *P* < 0.001 compared with the indicated group. SS, *Sargassum siliquastrum*; LPS, lipopolysaccharide; NO, nitric oxide.

**Figure 2:** SS extract inhibits LPS-induced iNOS expression by inducing heme oxygenase-1. (a) Real-time analyses to determine changes in mRNA levels of LPS-induced *Nos2* expression following treatment with the SS extract (SS). (b) Western blot analysis showing changes in the iNOS protein expression following the SS extract (SS) treatment. Densitometric analysis was performed using ImageJ software. The bars represent the mean ± standard deviation (SD); ^∗^: *P* < 0.05, ^∗∗^: *P* < 0.01, and ^∗∗∗^: *P* < 0.001 compared with the indicated group. SS, *Sargassum siliquastrum*; LPS, lipopolysaccharide; iNOS, inducible nitric oxide synthase.

The article "Ethanol Extract of Sargassum siliquastrum Inhibits Lipopolysaccharide-Induced Nitric Oxide Generation by Downregulating the Nuclear Factor-Kappa B Signaling Pathway" was published in 2022. Journal: Evid Based Complement Alternat Med.

**Figure 3:** SS extract inhibits LPS-induced proinflammatory cytokine expression and production. (a) Real-time PCR analyses to determine changes in mRNA levels of *Il1b*, *Il6*, and *Tnf* following treatment with the SS extract (SS) in LPS-stimulated RAW 264.7 cells. (b) ELISA to determine changes in the production of IL-6 and TNF-*α* following treatment with the SS extract in LPS-stimulated RAW 264.7 cells. The bars represent the mean ± standard deviation (SD); ^∗^: *P* < 0.05, ^∗∗^: *P* < 0.01, and ^∗∗∗^: *P* < 0.001 by comparison with the indicated group. SS, *Sargassum siliquastrum*; LPS, lipopolysaccharide.

**Figure 4:** SS extract blocks LPS-mediated activation of NF-*κ*B. (a–c) Western blot analyses showing changes in the total and phosphorylated forms of components of NF-*κ*B and AP-1 signaling pathways in cells pretreated with specific inhibitors (a) or the SS extract (SS) (b, c) for 24 h and stimulated with LPS (1 *μ*g/mL) for 30 min. Densitometric analysis was performed using ImageJ software. (d) A reporter gene assay showing regulation of NF-*κ*B transcriptional activity by the SS extract in RAW 264.7 cells stimulated with LPS (1 *μ*g/mL) in the presence or absence of the SS extract for 6 h. The bars represent the mean ± standard deviation (SD); ^∗^: *P* < 0.05, ^∗∗^: *P* < 0.01, and ^∗∗∗^: *P* < 0.001 compared with the indicated group. SS, *Sargassum siliquastrum*; LPS, lipopolysaccharide; NF-*κ*B, nuclear factor kappa-light-chain-enhancer of activated B cells; AP-1, activator protein-1.

**Figure 5:** SS extract enhances LPS-induced activation of the Nrf2/HO-1 pathway. (a) Western blot analysis of the total and phosphorylated forms of Akt and HO-1 in cells treated for 20 h with the SS extract in the absence or presence of LPS stimulation (1 *μ*g/mL). Densitometric analysis was performed using ImageJ software. (b) Real-time PCR analysis to determine changes in mRNA levels of Hmox1 following treatment with the SS extract (SS) in LPS-stimulated RAW 264.7 cells. (c) A reporter gene assay showing regulation of Nrf2 transcriptional activity by the SS extract in RAW 264.7 cells stimulated with LPS (1 *μ*g/mL) in the presence or absence of the SS extract for 6 h (d) Determination of changes in cellular ROS levels after 20 hours of LPS (1 *μ*g/mL) stimulation in the absence or presence of the SS extract. (e) Schematic diagram for the mechanism underlying the anti-inflammatory effect of the SS extract through inhibition of the NF-*κ*B pathway activation and enhancement of the LPS-induced Nrf2/HO-1 pathway. The bars represent the mean ± standard deviation (SD); ^∗^: *P* < 0.05, ^∗∗^: *P* < 0.01, and ^∗∗∗^: *P* < 0.001 compared with the indicated group. SS, *Sargassum siliquastrum*; LPS, lipopolysaccharide.

The article "Ethanol Extract of Sargassum siliquastrum Inhibits Lipopolysaccharide-Induced Nitric Oxide Generation by Downregulating the Nuclear Factor-Kappa B Signaling Pathway" was published in 2022. Journal: Evid Based Complement Alternat Med.

**Table 1:** Primer sequences used in this study.

Gene	Forward sequence (5′-3′)	Reverse sequence (5′-3′)
Nos2	CAGCTGGGCTGTACAAACCTT	CATTGGAAGTGAAGCGTTTCG
Il1b	AACCTGCTGGTGTGTGACGTTC	CAGCACGAGGCTTTTTTGTTGT
Il6	CTGCAAGTGCATCATCGTTGTT	CCGGAGAGGAGACTTCACAGAG
Tnf	CAGCCGATGGGTTGTACCTT	TGTGGGTGAGGAGCACGTAGT
Hmox1	AGGTACACATCCAAGCCGAGAA	CTCTGGACACCTGACCCTTCTG
Rn18s	GGAATAATGGAATAGGACCG	TCTGTCAATCCTGTCCGTGTCC

**Table 2:** Fatty acid contents in the SS extract.

Fatty acids	Amount (mg/100 g of SS extract)
Myristic acid (C14 : 0)	5.93
Pentadecylic acid (C15 : 0)	0.60
Palmitic acid (C16 : 0)	70.92
Margaric acid (C17 : 0)	0.87
Stearic acid (C18 : 0)	2.96
Behenic acid (C22 : 0)	2.09
Tricosanoic acid (C23 : 0)	52.77
Lignoceric acid (C24 : 0)	1.03
Total saturated fatty acids	137.17
Palmitoleic acid (C16 : 1)	6.07
Oleic acid (C18 : 1n9c)	18.93
Cis-11-eicosenoic acid (C20 : 1n9)	0.46
Erucic acid (C22 : 1n9)	0.43
Total monounsaturated fatty acids	25.89
Linoleic acid (C18 : 2n6c)	13.36
g-Linoleic acid (C18 : 3n6)	0.71
a-Linoleic acid (C18 : 3n3)	20.91
Cis-8,11,14-eicosatrienoic acid (C20 : 3n6)	2.38
Cis-11,14,17-eicosatrienoic acid (C20 : 3n3)	0.61
Arachidonic acid (C20 : 4n6)	0.40
Cis-13,16-docosadienoic acid (C22 : 2)	2.28
Cis-5,8,11,14,17-eicosapentaenoic acid (C20 : 5n3)	19.95
Cis-4,7,10,13,16,19-docosahexaenoic acid (C22 : 6n3)	0.51
Total polyunsaturated fatty acids	61.10
Total fatty acids	224.17

## Data Availability

All data generated or analyzed during this study are included in this published article.
